The article "Assessment of cognitive–motor functions in adults with perceived neuropsychological problems using NIH toolbox after remote biofield energy treatment as non‐pharmacological intervention: A randomized double‐blind placebo controlled trial" was retracted in 2026. Reasons: duplicate publication; overlap with earlier publications; unreliable results or conclusions; concerns about the data.

# Assessment of cognitive–motor functions in adults with perceived neuropsychological problems using NIH toolbox after remote biofield energy treatment as non‐pharmacological intervention: A randomized double‐blind placebo controlled trial

**DOI:** 10.1002/npr2.12482

**Published:** 2024-09-13

**Authors:** Mahendra Kumar Trivedi, Alice Branton, Dahryn Trivedi, Sambhu Mondal, Snehasis Jana

**Affiliations:** ^1^ Trivedi Global, Inc., Research and Development Henderson Nevada USA; ^2^ Trivedi Science Research Laboratory Pvt. Ltd., Research and Development Thane Maharashtra India

**Keywords:** biofield energy therapy, cognition–motor function, neuropsychological impairments, NIH toolbox, non‐pharmacological intervention, randomized clinical trial

## Abstract

Non‐pharmacological interventions include physical activity, biofield energy therapy, reiki, Tai chi, and therapeutic touch. However, no reports analyzed the effectiveness of biofield therapy on cognition and motor function performance in adult subjects. The study aimed to investigate the impact of remote biofield energy healing therapy on cognition and motor functioning in adults with self‐perceived neuropsychological impairments. This was a randomized double‐blind clinical trial that involved 114 participants with self‐perceived neuropsychological impairments. The participants were divided into three groups (control, sham control, and biofield intervention). Cognitive and motor function scores were assessed using the NIH Toolbox at baseline (day 0), day 90, and day 180. The biofield treatment group showed significant improvements in language function (*p* < 0.0001), working memory (*p* < 0.0001), and episodic memory (*p* < 0.0001) scores. Other cognitive functions also improved, although not statistically significant. The biofield intervention group also demonstrated significant enhancements (*p* < 0.05 to *p* < 0.0001) in locomotion, standing balance, dexterity, grip strength, and muscle endurance. No adverse effects were reported. The results suggest that remote biofield energy therapy is a safe, noninvasive intervention that improves cognitive and motor functions in adults. Further research is needed to understand its clinical benefits.

## Abstract 2

The remote biofield energy therapy resulted in significant improvements in cognitive and motor functions for the treatment group compared to the control groups, who received either no treatment or a sham treatment. This led to an overall improvement in neuropsychological functions and quality of life. The observed effects may be attributed to the healer's quantum thinking and the transmission of quantum energy therapy to the subjects at the quantum level through quantum entanglement.

## 1 INTRODUCTION

Cognitive and neuropsychiatric symptoms are common manifestations of various disorders.^1^ People with neuropsychiatric problems report a range of difficulties with concentrating, making decisions, slowed thinking, and forgetfulness. These symptoms reflect one of the core symptoms of these disorders.^2^ Numerous studies have also reported poorer neuropsychological performance on tests of memory, attention, and executive function in adults with stress, anxiety, and depression.^3^ These cognitive challenges can have a severe impact on patients' daily activities. Neurocognitive deficits are considered to be one of the criteria for attention deficit hyperactivity disorder (ADHD). Additionally, research has found links between these deficits, day‐to‐day function, and quality of life.^4^ The treatment options for providing benefits to patients with stress, anxiety, ADHD, depression, and cognitive deficits are limited. Most pharmacologic treatments provide little or nonsignificant benefit for cognitive impairment in neuropsychological symptoms, suggesting that non‐pharmacological interventions are needed to target cognitive–motor function impairments.^5^, ^6^, ^7^ Recently, biofield energy intervention, a non‐pharmacological therapy, showed significant positive effects on enhancing cognitive and motor functions in many studies.^8^, ^9^

Each life form has a biofield. The term “biofield” refers to the energy and materials that surround and permeate the human body. This energy controls the integrity of all organisms; controlling physical and biochemical reactions.^10^ The biofield energy therapies have many names such as Reiki, therapeutic touch, healing touch, acupuncture, Tai Chi, blessing, and external Qigong.^11^ This therapy is an energy therapy that involves the use of energy that flows naturally from the hands of the practitioner to the individuals to strengthen the body's ability to heal itself and thereby increase well‐being. It is reported to be a low‐risk, less‐expensive, noninvasive, easy‐to‐apply method that improves well‐being in many areas, such as decreasing anxiety,^12^ stress,^13^ psychological problems,^8^, ^12^, ^14^, ^15^ depression,^1^, ^2^, ^12^ cancer pain,^16^ arthritic pain,^17^ fibromyalgia,^18^ and improving cognition,^5^ attention and memory,^19^, ^20^ and quality of life.^14^, ^15^, ^21^ Biofield therapies have shown promising therapeutic benefits in treating various health disorders. With the increasing interest in complementary and alternative medicine (CAM) around the world, biofield therapies can be seen as a viable alternative therapy as non‐pharmacological intervention in clinics. Distant healing intention (DHI) is a popular form of CAM involving remote biofield energy therapy (RBET). Remote biofield energy therapies are intentional ways of healing that go beyond traditional space and time limitations and are believed to benefit clients' health. Numerous studies have shown evidence of DHI's successful healing effects.^22^, ^23^

The NIH Toolbox is used to assess neurological and behavioral functions to provide a brief, efficient, and highly accessible test to measure cognitive and emotional health.^24^ The NIH Toolbox divides tests into four domain batteries: cognition, motor, sensation, and emotion.^25^ The NIH Toolbox Cognition Battery (NTCB) was designed to assess key functions (language, processing speed, working memory, episodic memory, executive function, and attention) across the life span (age, 3–85 years). This computerized approach provides an economical method for assessing a wide range of cognitive abilities.^26^ Motor function and muscle movements are integrally related to daily activities and quality of life. Motor function is a complex physiological process and requires the integration of multiple inputs and systems, including the neuromuscular, neurosensory, musculoskeletal, and cardiopulmonary systems. Impairments in motor function often indicate central or peripheral nervous system disorders.^27^ Working memory is required for a wide variety of cognitive skills, such as long‐term memory, learning, reasoning, problem‐solving, planning, and active listening. Impaired working memory is common in medical disorders with neurological involvement, such as multiple sclerosis, traumatic brain injury, HIV, and schizophrenia.^20^ Language develops rapidly over the first 3 years of life. However, further changes occur throughout childhood, and language proficiency is a fundamental skill that supports many other aspects of cognitive, social, and behavioral function. Vocabulary has been used as a surrogate measure for overall crystallized intelligence. Oral reading proficiency is also a marker of educational opportunity in minority populations and can be used to adjust for group differences when comparing individuals of different ethnic and racial backgrounds.^28^ The subdomains of executive function deficits are seen in patients with acquired focal damage. In children, impairments in executive function or delays in its development have been linked to attention deficit hyperactivity disorder, autism spectrum disorders, conduct disorder, and other psychiatric conditions and symptoms.^29^ The subdomain processing speed is defined as either the amount of time it takes to process a set amount of information or the amount of information that can be processed within a particular unit of time. Simple processing speed tasks require a simple motor response to a target stimulus, while complex processing speed requires more concentration with some mental manipulation.^30^ Biofield therapy has been recognized as an alternative treatment by the National Institutes of Health since 1994. Practitioners often use their hands to deliver a steady flow of energy to the patient, either directly or virtually. This therapy was effective in reducing pain and discomfort in those with cancer, chronic pain, fatigue, and anxiety, as well as improving overall health.^14^, ^15^ However, it is worth noting that no study currently suggests that biofield energy therapy can improve cognition–motor function performance in healthy adults or patients with cognitive impairments. This paper aimed to evaluate the effect of remote biofield energy treatment as non‐pharmacological intervention therapy via remote (virtual) mode in adult subjects for the benefits of neuropsychological functioning and quality of life. Neuropsychological outcomes were assessed using cognitive and motor subsets of the NIH Toolbox.

## 2 MATERIALS AND METHODS

### 2.1 Study design

This study involved a randomized, placebo‐controlled, double‐blind, three parallel‐group, single‐center trial. The study was performed as per the ethical principles with good clinical practices from the Declaration of Helsinki.^31^ The clinical study protocol, informed consent document, and all other relevant study documentation were reviewed and approved by the Institutional Ethics Committee (IEC) of Riddhi Medical Nursing Home, Gujarat, India (ECR/886/Inst/GJ/2016/RR‐19). This study was approved by Clinical Trials Registry—India (CTRI) with clinical trial registration number—CTRI/2022/07/043943. A total of 173 subjects were screened, and 132 subjects meeting eligibility criteria were enrolled (1:1:1 ratio) in order to achieve 114 completed subjects (Figures 1 and 2).

**FIGURE 1:** Schematic diagram of study design.

**FIGURE 2:** The CONSORT flowchart representation of subject disposition.

### 2.2 Randomization procedure

After evaluation of screening parameters, receipt of a signed informed consent, and order of the investigational therapy for each subject, equal allocation of the sequence was ensured. The eligible subjects randomly assigned to the three groups, namely, control, sham control, and intervention group (1:1:1) with the help of a simple randomization technique (allocation concealment mechanism) using SAS software (Version: 9.4; SAS®, USA) to generate the random allocation sequence. The randomization schedule was maintained under controlled access. The personnel involved in distributing investigational therapy was accountable for ensuring compliance with the randomization schedule.

### 2.3 Blinding

This study was double‐blind, meaning that the treatments were blinded to the subjects and principal investigator/physician. In this study, the biofield energy treatments were done remotely for the participants on days 0 and 90. However, the staff involved in laboratory procedures and collecting objective data were blinded to the subjects under evaluation to maintain the study's integrity.

### 2.4 Sample size justification

A power analysis used to determine the sample size needed for the study. The researchers predicted a Cohen's *d* effect size of 0.8 for the treatment group. They estimated that 105 participants, accounting for a 10% drop‐out rate, would be needed to achieve a power of 80% and a type 1% error rate (alpha) of 5%. SAS software was used to assign the enrolled participants into three groups.

### 2.5 Inclusion criteria

The South Asian population (India; male and female) aged 20–55 years who met all the following criteria were included as appropriate participants in the trial, such as those who were 20–55 years old at the time of written informed consent. Subjects with a complaint with at least one or more neuropsychological symptoms (tiredness, fatigue, stress, anxiety, cognition impairment, poor memory, poor attention, emotional trauma, confusion, mental restlessness, mind chattering, lack of self‐worth, future/ongoing negative thoughts, etc.) were included in this trial. Body mass index (BMI) should be 18.5–35.0 kg/m^2^, calculated as weight in kg/(height in meters). Females of childbearing age agreed to use an acceptable form of birth control during the study. Agreed to provide written informed consent and able to follow the study directions to participate in the study and complete all follow‐up. Agreed to comply with the study requirements and procedures as per study protocol. Prior to enrolment, all subjects were screened by the principal investigator and physician for eligibility.

### 2.6 Exclusion criteria

Any participant met any of the following criteria was ineligible as (a) past history within last year or currently having alcohol dependence or drug abuse; (c) significant diseases or clinically significant abnormal findings in medical history, physical examination, laboratory evaluations, etc., during screening; (d) regular vigorous aerobic/endurance exercise (>3 vigorous bouts/week); (e) known history of positive HIV, HCV, HBsAg, or VDRL/RPR; (f) subjects with non‐healthy, non‐homogenous, damaged over the skin; (g) subjects with birthmarks or excessive hair over the skin; (h) subjects with the usage of self‐tanning agents for at least 10 days before screening; (i) female subjects who demonstrate a positive pregnancy test or currently breast‐feeding or planning pregnancy.

### 2.7 Withdrawal criteria

The investigator had right to withdraw a subject from the study for any of the following reasons: (a) if the subject withdrew his or her self‐consent for any reason; (b) if the subject's condition had worsened to the degree that the investigator feels, it was unsafe for the subject to continue in the study; (c) if the subject has taken any medication; (d) if an adverse event occurred for which the subject desired to discontinue treatment or the investigator determined that it was in the subject's best interest to be discontinued; (e) if there was any types of significant protocol deviation; (f) if a concomitant therapy was reported or required which was liable to interfere with the results of the study; (g) if the subject was lost to follow up; and (h) administrative reasons.

### 2.8 Biofield intervention strategy

The eligible subjects were assigned to the control (no intervention), sham control (sham healer's intervention), and biofield intervention/treatment group. The biofield intervention group subjects received two sessions of distant/remote biofield energy attunements (blessing/prayer) by an experienced (>15 years), renowned spiritual healing practitioner on day 0 and day 90, under the standard clinical laboratory setting. Briefly, the Biofield Energy Healing Therapy/Blessing Therapy was provided by the healing practitioner remotely from Florida, United States of America, via an online web‐conferencing platform (virtual mode) for about 5 min through his unique inherent thought transmission process (channeling universal life force energy) via laying his hands to the biofield intervention group of volunteers presented at Cliantha Research Limited, Ahmedabad, Gujarat, India. The start and end times of blessing therapy were recorded in the electronic case report forms (eCRF).

### 2.9 Assessment of cognitive and motor functions using NIH‐Toolbox test battery

All cognitive and motor assessments were administered by the trained investigator using the NIH Toolbox® Cognition/Motor Battery (NIHTB‐CB/MB, Version 1.25.6068) application.^32^, ^33^, ^34^, ^35^, ^36^ The subdomain structure was selected as per protocol. Through this process, six subdomains were identified as the most relevant areas of cognition functioning: language, processing speed, working memory, episodic memory, executive function, and attention. Moreover, five subdomains were identified as the most relevant areas of motor functioning: locomotion, standing balance, dexterity, grip strength, and endurance. Tests performed to assess the cognition and motor functions along with their score selected are presented in Table 1.

**TABLE 1:** The NIH‐Tool box recommended various standard tests were performed to assess the cognition and motor function along with their selected score.^24^

Type of activity	Test applied	Score selected
*Cognition core measures*		
Language	NIH Toolbox picture vocabulary test age 3+ v2.1	Age‐corrected standard score
Processing speed	NIH Toolbox pattern comparison processing speed test age 7+ v2.1	Age‐corrected standard score
Working memory	NIH Toolbox list sorting working memory test age 7+ v2.1	Age‐corrected standard score and fully corrected score
Episodic memory	NIH Toolbox picture sequence memory test age 8+ Form A v2.1	All three types of scores were used preferably the uncorrected standard score
Executive function	NIH Toolbox dimensional change card sort test age 12+ v2.1	All three types of scores were used with the computed score
Attention	NIH Toolbox flanker inhibitory control and attention test age 12+ v2.1	All three types of scores were used with the computed score
*Motor core measures*		
Locomotion	NIH Toolbox 4‐m walk gait speed test age 7+ v2.0	Computed score
Standing balance	NIH Toolbox standing balance test age 7+ v2.0	Fully corrected *T*‐score
Dexterity	NIH Toolbox 9‐hole pegboard dexterity test age 3+ v2.0	Fully corrected *T*‐score for dominant and non‐dominant hand
Grip strength	NIH Toolbox grip strength test age 3+ v2.0	Fully corrected *T*‐score for dominant and non‐dominant hand
Endurance	NIH Toolbox 2‐min walk endurance test age 3+ v2.0	Fully corrected *T*‐score

### 2.10 Safety assessment

An adult population was selected in which chances of interference of concurrent diseases were very unlikely and various safety‐related parameters (adverse events, medical history, physical examination of vital signs) and laboratory assessment (hematology) were performed. Our previous publication had already established the safety profile of biofield energy treatment on the human population.^14^, ^15^ Safety was determined by monitoring adverse effects (AEs), which were classified using the latest version of MedDRA (Medical Dictionary for Regulatory Activities) terminology.^37^ A complete premedical history, including a complete review of all current and past diseases and their respective treatments, was taken prior to starting study therapy.

### 2.11 Physical examination of vital signs

Physical examination of vital signs such as blood pressure (Digital Pressure Meter, Omron Healthcare Co. Ltd., Vietnam), pulse rate (Digital Pressure Meter, Omron Healthcare Co. Ltd., Vietnam), respiratory rate, and body temperature (Digital Thermometer, Nureca Limited, USA) was performed at the time of screening, randomization (day 0), treatment (day 90), and at the end of treatment (day 180), in order to evaluate the adverse effects if any. Subjects were remained in a seated position for about 5 min before vital signs were obtained.

### 2.12 Hematological parameter

Various safety‐related hematological parameters such as erythrocyte sedimentation rate (ESR; mm/1 h), hematocrit (HCT; %), hemoglobin (g/dL), mean corpuscular hemoglobin (pg), mean corpuscular hemoglobin concentration (g/dL), mean corpuscular volume (fL), platelet count (10^6^/L), total RBC count (10^12^/L), and total WBC count (10^6^/L) in order to evaluate the adverse effects. All the hematological parameters were measured using Sysmex XN‐550 hematology analyzer, Sysmex Corporation—Japan.

### 2.13 Statistical analysis

Continuous variables were expressed by means, medians, and standard deviations (SDs) in the descriptive analysis of the sample. For continuous variables, one‐way repeated analysis of variance (ANOVA), and for categorical variables, Chi‐square was used to calculate the *p*‐value. The data were represented as mean ± standard deviation/standard error of mean (SEM) and subjected to statistical analysis. Statistical analysis of NIH‐TB‐CB/MB test score (prior correction from baseline, CFB) was performed, and the level of significance (*p*‐value) was determined using one‐way repeated measure RM‐ANOVA followed by post hoc analysis by Tukey's test with 95% confidence interval (CI) of the difference between treatment using SigmaPlot (v14.0). Statistical analysis of NIH‐TB‐CB/MB test score after CFB was performed, and the level of significance (*p*‐value) was determined using one‐way repeated measure analysis of covariance (RM‐ANCOVA) with 95% CI of the difference between treatment using SAS® 9.4 (SAS Institute Inc., Cary, USA). The *p* < 0.05 was considered statistically significant. The authors compared the average variability between the groups and took the ratio of the mean sum of squares (MSB) to the error (residual) of the mean sum of squares (MSE). That is, the *F*‐statistic was calculated as *F* = MSB/MSE. Stat analysis data were reported as (F(between groups degree of freedom, residual error degree of freedom) = *F*‐value, *p*‐value). The outcomes of participants, who were randomized and received at least one intervention, were carried out using the intention‐to‐treat (ITT) analysis. We compared the results of the ITT with that per‐protocol (PP) analysis to check whether the results were consistent or not. The statistical results of the ITT and PP population data were the same, and the data are considered reliable. Therefore, the results of the ITT analysis were reported in the manuscript.

## 3 RESULTS

### 3.1 Disposition of study subjects

A total of 173 subjects were screened; 132 subjects met the eligibility criteria, enrolled in the study, and received study intervention; and 114 subjects completed the study. Among these, 35 (18 male + 17 female) subjects were assigned to the control group; 40 (18 male + 22 female) subjects were assigned to the sham control group; and 39 (19 male + 20 female) subjects were assigned to the blessing treatment group and continued at the end of study. A total of 18 subjects were discontinued from the study during the study period. The reason for discontinuation in the control group was consent withdrawal by subject (5) and lost to follow up (5 subjects). Similarly, in the sham control group, the reason for discontinuation was consent withdrawal by subjects (2) and lost to follow up (1 subject), and in the blessing group was consent withdrawal by subjects (3), and lost to follow up (2 subjects) (Figure 2).

### 3.2 Demographic and baseline characteristics

The South Asian males and females age between 20 and 55 years were enrolled in the study. Demographic characteristics of study subjects were recorded. The mean age for the subjects enrolled in the control, sham control, and blessing group was 37.5, 35.6, and 32.5 years, respectively. The mean BMI index for the subjects enrolled in the control group, the sham control group, and the blessing group was 24.78, 25.37, and 24.86 kg/m^2^, respectively. The male and female subjects' percentage in the control group (48.89%; 51.11%), the sham control group (48.84%; 51.16%), and the blessing group (47.73%; 52.27%) was comparable. Most of the enrolled subjects were married (i.e., around 76.52%). No statistically significant difference observed for any demographic characteristics, for example, gender, height, weight, and BMI except for age (*p* = 0.0172) across study treatment groups (Table 2). The same demographic data were shown in another manuscript to clarify and understand the results.

**TABLE 2:** Summary of demographic and clinical baseline characteristics.

Demographic and baseline characteristics	Control (*N* = 45)	Sham control (*N* = 43)	Biofield energy therapy (*N* = 44)
Age (years)			
Mean ± SD	37.5 ± 7.15	35.6 ± 6.71	32.5 ± 7.78
Median	38.0	36.0	32.0
Min, max	21, 54	23, 49	20, 49
*p*‐Value: 0.0172			
Sex (*n* [%])			
Male	22 (48.89)	21 (48.84)	21 (47.73)
Female	23 (51.11)	22 (51.16)	23 (52.27)
*p*‐Value: 0.9924			
Race (*n* [%])			
South Asian	45 (100)	43 (100)	44 (100)
Other	0 (0)	0 (0)	0 (0)
*p*‐Value: NE			
Height (cm)			
Mean ± SD	158.5 ± 10.60	160.2 ± 11.25	158.1 ± 9.36
Median	159.0	162.0	158.0
Min, max	137, 182	138, 180	141, 178
*p*‐Value: 0.8103			
Weight (kg)			
Mean ± SD	61.894 ± 9.1568	65.285 ± 14.2811	61.888 ± 10.0537
Median	61.650	62.000	61.825
Min, max	43.45, 85.6	44.1, 93.5	37.1, 89.05
*p*‐Value: 0.4608			
BMI (kg/m^2^)			
Mean ± SD	24.78 ± 3.828	25.37 ± 4.512	24.86 ± 4.307
Median	24.50	24.30	24.65
Min, max	18.8, 32.2	18.8, 34.6	18.6, 34.8
*p*‐Value: 0.9191			
Marital status (*n* [%])			
Divorced	3 (6.67)	1 (2.33)	1 (2.27)
Married	34 (75.56)	38 (88.37)	29 (65.91)
Married but separated	1 (2.22)	1 (2.33)	2 (4.55)
Single	5 (11.11)	3 (6.98)	10 (22.73)
Widow	2 (4.44)	0 (0)	0 (0)
Widower	0 (0)	0 (0)	2 (4.55)
*p*‐Value: 0.1240			
Smoking history (*n* [%])			
Previous	0 (0)	0 (0)	0 (0)
Current	0 (0)	0 (0)	0 (0)
Never	0 (0)	1 (2.33)	0 (0)
*p*‐Value: NE			

*Note*: The percentages were based on number of subjects in the specified treatment arm. BMI = weight (kg)/height (m^2^). For continuous variables, the *p*‐value was calculated by using one‐way analysis of variance (ANOVA) and for categorical variables, the *p*‐value was calculated by using the chi‐square test.

Abbreviations: BMI, body mass index; cm, centimeter; kg, kilogram; Max, maximum; Min, minimum; *n*, number of subjects in the specified category; *N*, number of subjects in the specified treatment arm; NE, not estimable; SD, standard deviation.

### 3.3 Assessment of cognitive–motor function before baseline correction using NIH toolbox

All the parameters were compared between the groups. Figure 3 presents the raw mean score (before correction from the baseline values) of all the cognitive and motor function parameters. It was observed that there was no significant difference between control versus sham control group (Figure 3).

**FIGURE 3:** The NIH toolbox (NIH‐TB) raw mean scores (prior correction from baseline, CFB) for cognitive and motor parameters are presented at day 90 and day 180, followed by various standard tests applied as per Table 1. The cognition domain measures are shown as (A) language, (B) processing speed, (C) working memory, (D) episodic memory, (E) executive function, and (F) attention. Moreover, motor domain measures are represented as (G) locomotion, (H) standing balance, (I) dexterity, and (J) endurance. Day 0 considered as the baseline. Statistical significance *p*‐value was calculated for between‐group comparisons using one‐way repeated measure analysis of variance (RM‐ANOVA) and for post hoc analysis was performed by Tukey's test. *p < 0.05, **p < 0.01, ***p < 0.001 show statistical significance versus control group; ^#^ *p* < 0.05, ^##^ *p* < 0.01, ^###^ *p* < 0.001 show statistical significance versus sham control group.

#### 3.3.1 Assessment of cognitive function

There was a statistically significant difference in cognitive measures, language score in the biofield intervention group at day 90 (*F*(2, 72) = 12.261, *p* < 0.001) and day 180 (*F*(2, 72) = 21.512, *p* < 0.001); processing speed at day 90 (*F*(2, 72) = 4.309, *p* = 0.024) and day 180 (*F*(2, 72) = 5.538, *p* = 0.007); episodic memory score at day 90 (*F*(2, 72) = 13.772, *p* < 0.001) and day 180 (*F*(2, 72) = 25.299, *p* < 0.001); executive function score at day 90 (*F*(2, 72) = 5.242, *p* = 0.017) and day 180 (*F*(2, 72) = 8.832, *p* < 0.001); and working memory function at day 90 (*F*(2, 72) = 34.860, *p* < 0.001) and day 180 (*F*(2, 72) = 38.543, *p* < 0.001) compared to the control group. Moreover, language score at day 90 (*F*(2, 72) = 12.261, *p* = 0.036) and day 180 (*F*(2, 72) = 21.512, *p* < 0.001); episodic memory score at day 90 (*F*(2, 72) = 13.772, *p* = 0.005) and day 180 (*F*(2, 72) = 25.299, *p* < 0.001); and working memory function at day 90 (*F*(2, 72) = 34.860, *p* < 0.001) and day 180 (*F*(2, 72) = 38.543, *p* < 0.001) were significantly improved in the biofield intervention group compared to the sham control group. Attention score did not show any significant changes (Figure 3A–F).

#### 3.3.2 Assessment of motor function

Motor domain measure of locomotion score was statistically significant in the biofield intervention group at day 90 (*F*(2, 72) = 17.535, *p* < 0.001) and day 180 (*F*(2, 72) = 35.924, *p* < 0.001); standing balance score at day 180 (*F*(2, 72) = 5.725, *p* = 0.005); endurance scores at day 180 (*F*(2, 72) = 11.796, *p* < 0.001); dexterity score at day 180 (*F*(2, 72) = 12.828, *p* < 0.001) compared to the control group. The locomotion score at day 90 (*F*(2, 72) = 17.535, *p* = 0.011) and day 180 (*F*(2, 72) = 35.924, *p* < 0.001) and dexterity score at day 90 (*F*(2, 72) = 3.478, *p* = 0.036) and day 180 (*F*(2, 72) = 12.828, *p* < 0.001) were significantly improved in the biofield intervention group compared to the sham control group (Figure 3G–J).

### 3.4 Assessment of cognitive–motor function after baseline correction using NIH toolbox

#### 3.4.1 Assessment of cognitive function

The mean score (after correction from baseline, CFB) of cognitive domain parameters such as language function was significantly increased from baseline to post‐intervention in the biofield intervention group at day 90 (*p* < 0.0001) and day 180 (*p* < 0.0001); working memory at day 90 (*p* = 0.0012) and day 180 (*p* < 0.0001); and episodic memory function at day 90 (*p* < 0.0001) and day 180 (*p* < 0.0001) compared to the control group. Moreover, the mean score of language function at day 90 (*p* = 0.0315) and day 180 (*p* < 0.0001); working memory at day 90 (*p* < 0.0001) and day 180 (*p* < 0.0001); and episodic memory function at day 90 (*p* = 0.0024) and day 180 (*p* < 0.0001) were statistically significant in the biofield intervention group with respect to the sham control group. Cognitive functions like language (*p* = 0.0278) and executive function (*p* = 0.0439) were significantly improved in the sham control group at day 90 compared to the control group. The processing speed, executive function, and attention mean scores were changed in the biofield intervention group as compared to the control as well as the sham control group; however, data were nonsignificant (Table 3).

**TABLE 3:** NIH toolbox (NIH‐TB) cognition–motor domain fully adjusted score after correction from baseline (CFB).

Parameter	Control (*N* = 35)		Sham control (*N* = 40)		Biofield energy therapy (*N* = 39)	
	Day 90 (mean^$^ ± SD)	Day 180 (mean^$^ ± SD)	Day 90 (mean^$^ ± SD)	Day 180 (mean^$^ ± SD)	Day 90 (mean^$^ ± SD)	Day 180 (mean^$^ ± SD)
*Cognitive function*						
Language	−0.2 ± 12.78	−3.5 ± 15.31	5.9 ± 11.52*	−2.2 ± 15.45	10.8 ± 10.73****/^#^	12.2 ± 12.12****/^####^
Processing speed	4.4 ± 8.69	4.9 ± 6.76	5.7 ± 10.37	6.4 ± 11.08	3.6 ± 6.91	4.5 ± 6.95
Working memory	2.3 ± 3.84	1.6 ± 2.23	1.5 ± 2.33	1.7 ± 2.52	2.8 ± 3.02**/^####^	4.4 ± 4.43****^/####^
Episodic memory	4.20 ± 59.36	13.60 ± 58.95	23.57 ± 57.21	29.69 ± 78.55	63.48 ± 77.89****/^##^	109.21 ± 89.76****/^####^
Executive function	0.12 ± 1.69	0.51 ± 1.70	0.53 ± 2.17*	0.68 ± 1.69	0.31 ± 1.95	0.70 ± 2.28
Attention	0.19 ± 1.12	0.32 ± 1.27	0.48 ± 1.03	0.32 ± 0.89	0.25 ± 0.86	0.17 ± 0.87
*Motor function*						
Locomotion	0.07 ± 0.32	0.06 ± 0.24	0.17 ± 0.29*	0.002 ± 0.28	0.29 ± 0.34****/^#^	0.39 ± 0.38****/^####^
Standing balance	−3.0 ± 13.25	−0.1 ± 9.87	2.6 ± 10.58	3.0 ± 11.66	−1.1 ± 14.91	5.5 ± 9.40*/^#^
Dexterity	1.4 ± 9.96	0.8 ± 6.87	0.8 ± 7.96	0.3 ± 8.12	1.5 ± 12.48	6.0 ± 10.90**/^####^
Grip strength	21.7 ± 14.34	17.2 ± 12.55	15.7 ± 12.13*	18.1 ± 10.51	19.4 ± 9.29	27.0 ± 10.61****/^###^
Endurance	−1.2 ± 8.17	−2.8 ± 6.84	0.2 ± 7.20	−2.6 ± 8.03	1.6 ± 7.43*/^#^	0.1 ± 6.22*/^###^

*Note*: All the values are represented as mean ± SD of CFB (change from baseline); ^$^CFB = (post baseline – baseline); *N* = number of subjects in the respective treatment group. Day 0 considered as the baseline. Statistical significance *p*‐value was calculated for between comparison using one‐way repeated measure analysis of covariance (RM‐ANCOVA). *p < 0.05, **p < 0.01, ****p < 0.0001 vs. control group; ^#^ *p* < 0.05, ^##^ *p* < 0.01, ^###^ *p* < 0.001, ^####^ *p* < 0.0001 versus sham control group.

#### 3.4.2 Assessment of motor function

The mean score of the motor domain parameters such as locomotion function was significantly improved from baseline to post‐intervention in the biofield intervention group at day 90 (*p* < 0.0001) and day 180 (*p* < 0.0001); standing balance at day 180 (*p* = 0.0113); dexterity at day 180 (*p* = 0.0015); grip strength at day 180 (*p* < 0.0001); and endurance at day 90 (*p* = 0.0333) and day 180 (*p* = 0.0268) compared to the control group. Moreover, mean score of locomotion function at day 90 (*p* = 0.0315) and day 180 (*p* < 0.0001); standing balance at day 180 (*p* = 0.0250); dexterity at day 180 (*p* = 0.0001); grip strength at day 180 (*p* = 0.0002); and endurance at day 90 (*p* = 0.0286) and day 180 (*p* = 0.0010) were significantly improved in the biofield intervention group compared to sham control group. Motor functions like locomotion (*p* = 0.0315) and grip strength (*p* = 0.0268) were significantly improved in the sham control group at day 90 compared to the control group (Table 3).

Based on the within‐group analysis, a slight difference was observed in the mean score of cognition–motor function (between baseline and day 90/180) of some parameters (processing speed, working memory, grip strength). However, those differences were insignificant in the control or sham control group. Moreover, significant differences (*p* < 0.05 to *p* < 0.001) were found in the cognition–motor function mean score between baseline and day 90 and 180 of parameters like standing balance, dexterity, episodic memory, executive function, language, locomotion, processing speed, working memory, grip strength in the biofield intervention group.

### 3.5 Safety assessment

No adverse effects (AEs) were reported during physical examination and the entire study period. No clinically significant vital signs finding was observed during the study (Table 4). The hematological test results were within the normal range at baseline and follow‐up (Table 5).

**TABLE 4:** Assessment of vital signs.

Vital sign	Control (*N* = 45)			Sham control (*N* = 43)			Biofield energy therapy (*N* = 44)		
	Day 0 (mean ± SD)	Day 90 (mean ± SD)	Day 180 (mean ± SD)	Day 0 (mean ± SD)	Day 90 (mean ± SD)	Day 180 (mean ± SD)	Day 0 (mean ± SD)	Day 90 (mean ± SD)	Day 180 (mean ± SD)
SBP (mmHg)	119.70 ± 11.15	119.30 ± 11.21	120.80 ± 11.93	115.50 ± 11.48	117.40 ± 11.24	123.00 ± 6.85	117.50 ± 11.06	115.60 ± 11.97	120.10 ± 9.63
DBP (mmHg)	76.7 ± 7.34	78.0 ± 6.99	78.1 ± 7.62	76.8 ± 7.96	76.8 ± 6.41	80.2 ± 5.91	75.8 ± 6.86	76.4 ± 7.51	79.1 ± 7.31
Pulse rate (beats/min)	79.3 ± 5.81	77.2 ± 7.62	77.9 ± 7.21	75.0 ± 7.30	79.2 ± 6.46	78.7 ± 5.57	80.3 ± 6.38	78.7 ± 6.99	78.9 ± 5.97
Respiratory rate (breath/min)	15.4 ± 1.88	15.3 ± 1.63	15.1 ± 1.42	15.0 ± 1.98	15.1 ± 1.64	14.8 ± 1.33	15.3 ± 1.80	15.3 ± 1.64	14.9 ± 1.42
Body temperature (°F)	97.32 ± 0.61	97.58 ± 0.55	97.17 ± 0.60	97.53 ± 0.50	97.45 ± 0.65	97.24 ± 0.38	97.22 ± 0.62	97.45 ± 0.49	97.22 ± 0.37

Abbreviations: DBP, diastolic blood pressure; SBP, systolic blood pressure.

**TABLE 5:** Assessment of hematological parameter.

Parameter	Control (*N* = 45)			Sham control (*N* = 43)			Biofield energy therapy (*N* = 44)		
	Day 0 (mean ± SD)	Day 90 (mean ± SD)	Day 180 (mean ± SD)	Day 0 (mean ± SD)	Day 90 (mean ± SD)	Day 180 (mean ± SD)	Day 0 (mean ± SD)	Day 90 (mean ± SD)	Day 180 (mean ± SD)
ESR (mm/1 h)	8.60 ± 2.67	8.70 ± 1.97	9.70 ± 1.64	8.70 ± 2.99	7.90 ± 2.57	10.20 ± 1.75	10.60 ± 1.85	8.70 ± 2.81	10.20 ± 1.64
HCT (%)	39.39 ± 4.19	40.19 ± 5.08	38.83 ± 4.36	39.08 ± 4.41	40.29 ± 5.19	38.22 ± 4.19	39.25 ± 4.24	40.70 ± 4.06	38.92 ± 4.13
Hb (g/dL)	12.54 ± 1.52	12.56 ± 1.82	12.11 ± 1.55	12.22 ± 1.64	12.31 ± 1.95	11.85 ± 1.59	12.59 ± 1.60	12.43 ± 1.47	12.22 ± 1.54
MCH (pg)	28.30 ± 4.14	27.41 ± 4.28	27.18 ± 4.06	26.83 ± 4.45	25.56 ± 4.17	25.16 ± 4.00	27.40 ± 3.48	25.99 ± 3.20	25.62 ± 2.91
MCHC (g/dL)	31.79 ± 1.30	31.18 ± 1.33	31.16 ± 1.13	31.23 ± 1.39	30.48 ± 1.44	30.93 ± 1.418	32.02 ± 1.211	30.50 ± 1.092	31.36 ± 1.232
MCV (fL)	88.79 ± 10.82	87.60 ± 11.09	87.01 ± 10.91	85.57 ± 11.30	83.57 ± 10.66	81.07 ± 10.03	85.42 ± 9.26	85.08 ± 8.80	81.61 ± 7.61
Platelet count (10^6^/L)	346 800.00 ± 93 617.84	337 473.70 ± 115 413.18	309 514.30 ± 80 008.22	319 046.50 ± 87 704.58	326 487.80 ± 84 980.33	323 225.00 ± 81 896.90	353 818.20 ± 91 881.69	339 463.40 ± 76 673.69	349 769.20 ± 84 475.30
Total RBC count (10^12^/L)	4.49 ± 0.64	4.64 ± 0.68	4.51 ± 0.64	4.63 ± 0.73	4.87 ± 0.72	4.78 ± 0.69	4.64 ± 0.62	4.82 ± 0.63	4.80 ± 0.57
Total WBC count with differential (10^6^/L)	7290.70 ± 2081.85	7196.30 ± 1875.15	7375.10 ± 2146.84	7063.30 ± 1640.36	7134.60 ± 1623.33	6869.00 ± 1681.36	7135.50 ± 1730.24	6719.30 ± 1793.46	7126.20 ± 1907.82

Abbreviations: ESR, erythrocyte sedimentation rate; Hb, hemoglobin; HCT, hematocrit; MCH, mean corpuscular hemoglobin; MCHC, mean corpuscular hemoglobin concentration; MCV, mean corpuscular volume; RBC, red blood cells; WBC, white blood cells.

## 4 DISCUSSION

The subjects with cognitive–motor function impairment had more difficulties performing routine tasks, leading to reduced participation in social activities and a reduced quality of life. There is insufficient evidence to support a pharmacological intervention with disease‐modifying therapies to improve cognitive and motor function.^38^ Moreover, in the last few years, the effects on cognition–motor function performance by other non‐pharmacological interventions like biofield energy treatments such as Reiki therapy, qui, therapeutic touch, healing touch, biofield therapy, and physical exercise were also studied and reported significant effects on the improvement of cognitive and motor function of neuropsychiatric disorders.^13^, ^16^, ^39^ Holistic therapy, like biofield energy therapy, is a more effective, side‐effect‐free, and less expensive treatment as compared to modern medicine. Biofield energy therapy has gained attention in recent years, and several studies have investigated its efficacy in treating psychosomatic disorders in adult subjects.^40^, ^41^ Distant (or distance) healing intention involves various forms of remote biofield energy therapy such as therapeutic touch, Reiki healing, external qigong spiritual healing, and prayer. It refers to a deliberate and conscious mental effort aimed at improving another person's physical or emotional well‐being from a distance.^42^ RBET claims to promote healing through exchanging or channeling energy beyond the physical realm. Therefore, this study has focused on multimodal treatment paradigms designed to target several cognition–motor domains using the NIH toolbox.

The NIH‐TB test battery is a widely applicable, brief, diverse, accessible, and psychometrically sound set of instruments for evaluating neuropsychological behaviors in a wide age range.^43^, ^44^ Authors did not find direct references that correlate the current study outcomes. Hence, the findings in this trial are correlated with similar reported studies. Reiki therapy improved memory problems in mild cognitive impairment and Alzheimer's patients.^45^ Tai Chi intervention improved memory and cognitive function in mild cognitive impairment people.^46^, ^47^ Qigong therapy significantly improved cognitive functions in cognitive impaired Chinese adults.^48^ The current trial results demonstrate that there was an improvement in the performance on the NIH‐TB cognition and motor functions as a result of biofield energy therapy administered remotely. The findings are scientifically sound, robust, validated, and consistent to draw a meaningful conclusion. This study provides the first comprehensive report with significant improvement of most cognitive and motor functions for assessing neuropsychological properties. We found that exposure to distance life force energy/remote biofield energy therapy can induce significant enhancements in cognitive performance in the study subjects. One publication reported that the therapy (RBET) effects could be due to the healer's quantum thinking and transmission of the quantum energy to the subject leads to the healing that occurs spiritually through instantaneous communication at the quantum level via quantum entanglement.^49^ The main improved cognitive test battery functions include language, working memory, and episodic memory in the biofield intervention group, while language and executive function were improved in the sham control group (Table 3). However, before CFB, all six cognitive function scores were significantly improved in the biofield intervention group (Figure 3). Cognitive function parameters, processing speed and attention showed marginal changes in sham control and biofield intervention groups as compared to the control group, but the data were not statistically significant (Table 3).

The motor function can integrate different physiological systems such as musculoskeletal, neuromuscular, cardiopulmonary, neural motor, and sensory‐perceptual systems. The motor–functional status is an indicative marker of current physical health status, disease burden, and future health outcomes and is ultimately related to daily functioning and quality of life.^24^, ^27^ This study evaluated the conceptual and clinical relevance of critical aspects of motor function (five subdomains) in the motor functions of the NIH Toolbox. Gait speed is a measure of bipedal locomotion that indicates the overall disease burden and prognosis in older persons. It also predicts the length of stay and discharge of patients admitted to rehabilitation centers after a stroke, incident dementia, etc.^50^ Assessment of standing balance is essential as it predicts people's ability to perform various daily activities safely and independently. Several studies have reported changes in balance ability that directly correlate with the changes in function.^51^ Dexterity is a central component of hand function that involves both speed and accuracy of hand movements while manipulating objects in the environment. Muscle strength is an essential component for humans to perform daily activities. The grip strength has been used to characterize total body strength and predict mortality, postsurgical complications, and future disability.^52^ Muscle endurance and cardiorespiratory are essential to physical fitness, performance, and health status. People with better endurance can complete daily tasks, high workloads, etc. In this study, two parameters (locomotion and endurance) at day 90 and all five motor function parameters at day 180 were significantly (*p* < 0.05 – *p* < 0.0001) improved in the biofield intervention group with respect to the control and sham control groups. Besides, locomotion and grip strength scores showed a significant (*p* < 0.05) difference in the sham control group compared to the control group (Table 3). Motor function parameter like attention showed marginal changes, but the data were not statistically significant (Figure 3).

The experimental design of the study is a strength of this work. The strengths also include the sensitivity and accuracy of datasets toward neuropsychological effects and their efficiency as authors utilized NIH Toolbox, a well scientifically computerized software‐based instrument. The results are statistically significant and very promising with respect to both cognitive and motor function. In addition to our findings, there are a few limitations: single‐center setting, a single type of population studied, lack of a reliable biofield energy measurement, lack of mechanism of actions of this therapy, ceiling effects on some tasks, floor effects, and variable measurement sensitivity to cultural/socioeconomic factors. Future work with multiple types of populations should clarify reliability and validity within individuals.

## 5 CONCLUSION

This is the first report where we present remote biofield energy therapy as a non‐pharmacological intervention that significantly improved most of the cognition–motor functions in the biofield intervention group in adult subjects with self‐perceived neuropsychological impairments. It was also found that a few parameters (language, executive function, locomotion, and grip strength) were significantly improved in the sham control group. This novel treatment approach may help to design and conduct future clinical studies with specific symptoms for managing neuropsychological disorders.

## FUNDING INFORMATION

The authors declare that no funds, grants, or other support were received during the preparation of this manuscript.

## CONFLICT OF INTEREST STATEMENT

MKT, AB, and DT were employed by Trivedi Global, Inc. SM and SJ were employed by Trivedi Science Research Laboratory Pvt. Ltd.

## ETHICS STATEMENT

Approval of the Research Protocol by an Institutional Reviewer Board: The study was conducted in accordance with the ethical principles originating from the Declaration of Helsinki and consistent with good clinical practices. The clinical study protocol, informed consent document, and all other relevant study documentation were reviewed and approved by the Institutional Ethics Committee (IEC) of Riddhi Medical Nursing Home, Gujarat, India (ECR/886/Inst/GJ/2016/RR‐19).

Informed Consent: Written informed consent was obtained from all the participants.

Registry and registration no. of the study/trial: This clinical trial study is registered in the Clinical Trials Registry – India (CTRI: CTRI/2022/07/043943).

Animal Studies: Not applicable.

## Supporting information


File S1.

## Data Availability

The raw datasets were given as supplementary file.
